# Do Coaches Perceive Themselves as Influential on Physical Activity for Girls in Organised Youth Sport?

**DOI:** 10.1371/journal.pone.0105960

**Published:** 2014-09-03

**Authors:** Justin M. Guagliano, Chris Lonsdale, Richard R. Rosenkranz, Gregory S. Kolt, Emma S. George

**Affiliations:** 1 School of Science and Health, University of Western Sydney, Sydney, Australia; 2 Institute for Positive Psychology and Education, Australian Catholic University, Sydney, Australia; 3 Department of Human Nutrition, Kansas State University, Manhattan, Kansas, United States of America; Tokyo Institute of Technology, Japan

## Abstract

Participation in organised youth sports (OYS) has been recommended as an opportunity to increase young peoples' physical activity (PA) levels. While coaches can potentially influence athletes' PA levels, what has not been explored is the question; do coaches perceive themselves as influential on PA for girls in OYS? Participants were 30 coaches of girls OYS teams aged 9–17 years in the Greater Sydney Metropolitan Area, Australia. Participants took part in a semi-structured interview that lasted approximately 30 minutes. They responded to questions regarding their perceived role as coaches, their perceptions of themselves as role models for PA, their views on their athletes' current PA levels, their opinions on improving their athletes' PA levels, and their perceived challenges as coaches in OYS. Many coaches considered themselves role models for PA due to their own involvement in organised sports. Coaches felt that they were conscious of girls' PA levels during training and could accurately gauge how active girls were. Coaches perceived their training sessions to provide sufficient PA and thus, did not feel the need to try to increase PA during training. Many coaches were cautious about conducting training sessions where the PA intensity was high for prolonged periods because they believed that it could potentially result in dropout from OYS. Coaches' perceived time commitment to OYS, variability of skill/experience amongst girls, and poor parental support as major challenges they experienced in OYS. This study provided a unique insight from the perspective of coaches in OYS. Most coaches felt that they had the potential to influence PA for girls in OYS; however, coaches may underestimate or not fully realise the impact they can have on the girls they coach. Future research should focus on educating coaches to capitalise on the opportunity they have to promote PA through OYS.

## Introduction

Organised youth sports (OYS) is a structured physical activity (PA) setting for children and adolescents that is governed by the rules of the sport being played [1]. In OYS, athletes attend training sessions and games under supervision of one or more adults, who most often assume the role of team coach [1], [2]. Coaches in OYS are in an ideal position to impact the health and well-being of children and adolescents. Due to their role in OYS, coaches can carry considerable influence, as they are viewed as experts by their athletes [3]. Similarly, Smith and Smoll [4] have suggested that coaches can have a strong impact on children and adolescents within an OYS context due to the amount of direct involvement they have with their athletes on a weekly basis. Coaches also have considerable reach, as high proportions of children and adolescents participate in OYS around the world [5]. The most recent prevalence data indicate that, approximately 66% of all Australian children (67% of all boys and 65% of all girls) participate in at least one OYS (including dance) outside of school hours [6], [7]. Through their participation in OYS, children and adolescents have the potential to be exposed to an array of physical and psychosocial health and developmental benefits [8]–[11].

Arguably, one of the most pertinent attributes of OYS is its potential to contribute significantly to moderate-to-vigorous physical activity (MVPA) levels of participating children [12], [13]. Children and adolescents should engage in at least 60 minutes of MVPA daily and vigorous PA, including activity that strengthens muscle and bone, should be incorporated at least three times per week [14]–[16]. However, since a sizeable proportion of children and adolescents around the world do not meet the recommended levels of daily MVPA [5]. In Australia, a recent report found that less than one-fifth of Australian children and adolescents, aged 5–17, met recommended physical activity guidelines every day of the week [6]. This issue is even more concerning when examining youth PA levels separately, by gender. Girls are less physically active than boys throughout childhood [17], [18] and their participation in PA declines more sharply than in boys as they transition into adolescence [17], [19]. As such, girls have been identified as a high priority group for PA promotion [20], therefore participating in OYS can have major public health implications. Although participation in OYS provides an ideal opportunity for children and adolescents to accumulate substantial amounts of MVPA, participation in OYS does not guarantee MVPA. Studies have found that children and adolescents spend large proportions of time during OYS inactive or in light PA [12], [21], [22]. Furthermore, coaches spent a considerable proportion of training time in management and knowledge delivery contexts [12], where it is likely that children and adolescents would be relatively inactive [23].

Coaches, therefore, have the opportunity to influence their athletes' PA levels, particularly during training where coaches are better able to dictate the intensity of PA, compared to a game. However, the way coaches perceive themselves with regards to influencing girls' PA is not clear and further exploration is warranted due to the high proportion of children who participate in OYS and the myriad of health and developmental benefits children and adolescents stand to gain through the setting. OYS presents a good opportunity to participate in PA and has the potential to be a powerful health-promoting environment for children and adolescents, where coaches are at the helm.

To our knowledge, no study has explored whether coaches perceive themselves as influential on PA for girls participating in OYS. Further, only a few cross-sectional studies have examined children and adolescents' PA levels in OYS [12], [21], [22], finding that children and adolescents spent large proportions of time during OYS inactive or in light PA. Coaches' views on their athletes' current PA levels and their opinions on improving their athletes' PA levels, however, have not been investigated. Lastly, coaches' perceived challenges in OYS have also not previously been considered, and as such, this information could provide valuable insight on aspects of the coaching experience that could inform future studies aiming to increase PA in OYS. Accordingly, this study aimed to explore OYS coaches': (1) perceived role as a coach; (2) perception of themselves as role models for PA; (3) views on their athletes' current PA levels; (4) opinions on improving their athletes' PA levels; and (5) their perceived challenges as coaches in OYS.

## Methods

### Study design and procedures

This study conforms to the consolidated criteria for reporting qualitative research (COREQ) developed by Tong, Sainsbury, and Craig [24]. Between July and August 2012, each of the 30 coaches recruited took part in one in-depth semi-structured interview with the primary author (JMG). Interviewing is one of the most commonly used methods in qualitative research [25] and is a method capable of providing rich and comprehensive data [26]. Semi-structured interviews also provide the interviewer with the flexibility to further explore participants' responses [27].

The interview questions, prompts, and probes used in this study are outlined in Table 1. The development of the interview questions was guided by the aforementioned study aims. Most interview questions were open-ended to elicit a wide range of responses and prompts and probes were used to encourage further discussion, when required. To ensure content validity, the interview guide was iteratively developed by all members of the research team; reviewing content, structure, and wording of the questions. The research team also assessed the ordering of the interview questions and length of the interview. The questions were pilot tested on three adults who had coaching experience in a range of sports to ensure appropriate face validity.

**Table 1:** Interview questions, prompts, and probes.

• How do you describe your role as a coach?
• In terms of physical active, do you see yourself as a role model for your athletes?
○ In relation to having a healthy/active lifestyle?
• In what ways do you think you can influence the health behaviours of your athletes?
• How active do you think the athletes are during training?
• Can you tell me about the major demands or challenges you face as a coach?
○ Personal (e.g., lack of time, work or family commitments)
○ Athletes (e.g., lack of motivation, interest, or discipline)
○ Parents
○ Facilities/equipment
• If you were asked to make changes to your team with regard to promotion of greater physical activity levels during training time, what factors would influence your ability to do that?
• How important is it to you that your athletes are physically active during training?
• Can you identify ways you could increase children's physical activity levels during organised sport training?
• How do you plan what you're going to do for a training session? Take me through your process.
• How important is it to you that your athletes are physically active outside of organised sport?
• To what degree do you think you are responsible for influencing the physical activity behaviours of your athletes outside of organised sport?

Each participant was informed that the current study would be disseminated as part of JMG's doctoral thesis and associated publications, and all participants provided verbal and written informed consent prior to participating in their interview. All interviews were conducted face-to-face, and the majority of the interviews took place at a training ground prior to one of the participants' regular scheduled training sessions (23/30 interviews). Interviews were also conducted at participants' homes (5/30) or at a local café (2/30 interviews), as these locations were most convenient for the coaches. Each interview was conducted in a private or semi-private location and only the participant and the primary author were present during the interviews. The interviews lasted approximately 30 minutes, ranging from 28–40 minutes. At the conclusion of each interview, the participant received a $50 gift card as compensation for their time. Following each interview, field notes were made by JMG reflecting any key moments or quotes that occurred.

All interviews were conducted by JMG, who has conducted prior research on the chosen organised sports [12]. He has four years of personal experience coaching childrens' organised sport teams, and has played soccer for over 20 years. JMG is also working towards a doctoral degree in the area of PA promotion in children and youth, and currently holds an honours bachelor's degree in community health sciences. This knowledge and experience of sports and coaching was useful, because it helped build rapport with participants, and ensured jargon used by the coaches was understood. Most participants did not have any prior relationship with the research team; however, five coaches were involved in a previous study [12].

### Participants

A convenience sample of OYS coaches who coached club and representative level teams of girls aged 9 to 17 years participated in this study. In this study, a club-level coach coaches athletes that have registered with an OYS club and have been assigned to a team. Representative athletes are also registered with an OYS club; however, these athletes were selected members of a team. Representative athletes represent their district and compete in a higher level of competition than club athletes. The representative-level is not the highest level of competition in OYS; however, higher levels of competition were not discussed in this study.

Participants were recruited from OYS clubs playing netball, basketball, and outdoor soccer (football) in the Greater Sydney Metropolitan Area, Australia. These organised sports were chosen because of their popularity amongst girls (in terms of participation rates) in Australia [28]. Initially, a member of each of the organised sport club's executive committee was contacted by the primary author (JMG), to provide information about the study. Clubs then provided contact details (a phone number and/or an email address) of interested participants who were coaching girls' teams in the appropriate age range. Detailed study information was then sent via email to each potential participant and coaches were included based on their willingness to participate in the study. The Human Research Ethics Committee of the University of Western Sydney approved this study.

Participant characteristics are detailed in Table 2. In total, 30 coaches (10 coaches from each of the three organised sports) participated. Coaches were aged 18–69 years (mean age = 42.2±13.2 years) and had an average of 13.3±11.8 years of coaching experience. The majority of the coaches were male (63%), married (57%), educated at a tertiary level (57%), held a form of coaching credential related to their sport (90%), and were overweight (43% with ≥25 BMI<30) or obese (30% with BMI≥30), based on participants' self-reported height and weight.

**Table 2:** Characteristics of Participating Coaches.

Variable	Netball	Basketball	Soccer
	(n = 10)	(n = 10)	(n = 10)
Mean age (±SD)	41.8(18.8)	38.8(12.3)	45.8(5.4)
Sex, n			
Male	2	8	9
Female	8	2	1
Mean height (cm) (±SD)	165.7(9.4)	179.3(11.4)	176.2(10.8)
Mean weight (kg) (±SD)	74.6(13.1)	83.3(20.2)	94.4(15.2)
Mean body mass index (±SD)	27.2(4.2)	25.6(4.3)	30.3(5.3)
Marital Status, n			
Married	4	5	8
Divorced	1	1	0
Not married	5	4	2
Level of education, n			
University or higher	2	3	1
Certificate/diploma	3	3	5
Trade/apprenticeship	1	0	1
Secondary school	3	2	2
Less than secondary school	1	2	1
Annual income, n			
$100,000+	3	2	7
$80,000–$99,999	1	5	1
$60,000– $79,999	1	0	1
$40,000–$59,999	2	0	1
$20,000–$39,999	0	2	0
<$20,000	3	1	0
Mean years coaching (±SD)	18.5(16.3)	12.8(8.7)	8.5(7.2)
Mean number of sports coaching (±SD)	1(0)	1.1(0.3)	1.5(0.9)
Mean number of age groups coaching (±SD)	1.8(0.6)	2.8(0.8)	1.7(1.0)
Coaches with coaching credentials, n	10	10	7

Note: n = number of coaches.

### Data analysis

Interviews were audio-recorded and transcribed verbatim by JMG. During transcription, further notes were added to the original field notes made during post-interview reflection. After transcription, 20% of transcripts were returned to corresponding participants for verification. To ensure equal representation, two participants (a male and a female) were selected from each sport for verification. Participants made no changes to their transcripts.

Using a long table approach, content analysis was conducted using guidelines established by Côté, Salmela, Baria, and Russell [29]. Due to the exploratory nature of this study, an interpretational approach to analysis was used [30]. Côté et al. [29], described two separate phases for interpretational qualitative analysis: (1) data organisation (or creating tags) and (2) data interpretation (or creating categories). The process used to analyse the data is illustrated in Figure 1. A decision-making heuristic for the analysis of unstructured qualitative data by Côté and Salmela [31] was also used.

**Figure 1:** Data analysis process.

During the data organisation phase, text from each transcript (and corresponding field notes) were divided into segments called meaning units to produce a set of concepts that reflected meaningful pieces of information [29]. Text was divided into meaning units directly on each transcript, where tags were assigned to each meaning unit. Tagging was performed by JMG. A separate document was kept as an inventory of all the accumulated tags for the second phase of the analysis. For the data interpretation phase, the inventory of tags from all transcripts was examined by JMG and ESG. For our purposes, a deductive process was used to underpin the coding framework and help organise tags; where tags fell within five overarching categories (the aims of this study). An inductive process, however, was used to group tags with similar meaning together, which led to the emergence of themes and sub-themes within each overarching category. Disagreements while categorising were discussed with two members of the research team (CL and GSK) until a consensus was reached.

Sample size was determined *a priori* to ensure equal representation of the three organised sports. Transcripts were analysed after all interviews were conducted, in the order in which the interviews were conducted to determine theoretical saturation. Côté et al. [29] stated that theoretical saturation is reached when new data fits adequately into the existing framework. Theoretical saturation was determined to have occurred following the 23^rd^ interview.

In order to assess classification consistency, a random sample of 25% of tags was selected for independent classification under mutually exclusive categories and themes by a member of the research team familiar with the study aims but removed from data analysis until this point (RRR). Agreement was determined by comparing RRR's independent classification of a random sample of tags with the classification of tags conducted by the rest of the research team. Seventy percent agreement was set as the minimum acceptable level of agreement. Agreement was also assessed using Cohen's kappa coefficient. RRR's independent classification of a random sample of tags showed a high level agreement with the rest of the research team (88.6% agreement, kappa coefficient = 0.88).

## Results

A summary of the main themes, sub-themes, and example quotes that emerged from the 30 in-depth semi-structured interviews with OYS coaches are presented by category in Tables 3 to 7. The five categories are presented in the following order: (1) participants' perceived role as coaches (five themes, three sub-themes); (2) their perception of themselves as role models for PA (two themes, no sub-themes); (3) their views on their athletes' current PA levels (five themes, no sub-themes); (4) their opinions on improving their athletes' PA levels (five themes, two sub-themes); and (5) their perceived challenges as coaches in OYS (four themes, nine sub-themes).

**Table 3:** Perceived role as coaches: summary of categories, themes, sub-themes, and example quotes.

Category	Themes	Sub-themes	Example quotes
Perceived role as a coach	Teacher	To foster sports-related development	“My main role is to teach them how to be better soccer players. I focus on developing their soccer skills, preparing them for games and keeping them focused” [SC 6].
		To foster the development of other life skills	“For the girls, I would hope I'm seen as kind of like a life coach. I try focus on teaching them things they can learn through sport that can be used later in life like I tell them if you lose a ball, you have to make sure you get back and try to win it back because you are not helping the team if you don't – that's being accountable” [SC 3].
		To create positive environment	“…I'm a bit of a joker at times and I try to keep the atmosphere as light, fun, and friendly as possible and I think I have a pretty good rapport with the kids” [NC 15].
	Role Model		“I see myself as a role model for the girls… I'm only a little bit older than the girls on my team and I want them to know that I don't care if other people judge me because I play sport and if they say things like ‘oh it's not girly to be running around playing sport getting sweaty’. I want to show them that it's just sports, I do it, and everyone should be doing it, really. [NC 17].
	Mentor		“I'm more of a mentor, someone who's guiding them to achieve the goals that they want and helping them develop the skills that they need to achieve those goals” [SC 10].
	Facilitator		“I organise their training sessions once a week, prepare them for the game… make sure they are ready to go, that they know what we're doing, adjusting positions, making sure everyone has equal court time… and I take care of all the paperwork.”[NC 16].
	Disciplinarian		“A lot of people will tell you I'm a meanie (laughs). So, I suppose I'm a disciplinarian because I'm strict.” [BC 20].

SC = soccer coach; NC = netball coach; BC = basketball coach.

**Table 4:** Coaches' perceptions of themselves as role models for physical activity: summary of categories, themes, sub-themes, and example quotes.

Category	Themes	Sub-themes	Example quotes
Coaches' self-perceptions as role models for athletes	Positive self-perception as a role model for physical activity		“They see me play on Monday nights in the men's comp and I train with them all the time, running around; so hopefully they see me as a role model both for basketball skills as well as the fitness aspect of it.” [BC 25].
			“I've never really thought about it, but yeah, I haven't not played sport (laughs)… and most of the kids that I coach know that I've played at a pretty high level too. So I'd consider myself a pretty good role model.” [BC 20].
			“I do because this is my lifestyle. I find it odd that people aren't physically active, you know (laughs). I'm a PE teacher, I coach, play, umpire, I'm in an old ladies representative team as well, so you know, it's just what I am about and hopefully some of that rubs off.” [NC 13].
			“…not only in the teams that I'm coaching but also in my general life with people around the netball courts. I'm definitely a role model to people around the netball courts in terms of longevity, how long can you do this sport? And people just sort of respect that I think.” [NC 8].
	Negative self-perception as a role model for physical activity		“…probably not in the physical activity sense – I'm a bit passed that… I'm not the fittest 50-year old I know.” [NC 15].
			“Probably not, you're talking to an old bugger here.” [SC 6].
			“Not since my knees have gone on me.” [BC 11].
			“Oh look, probably not. I don't actually play netball anymore, I did for 15 years previously, but my physical activity has sort of taken a dip.” [NC 16].

SC = soccer coach; NC = netball coach; BC = basketball coach.

**Table 5:** Coaches' perceived levels and importance of physical activity: summary of categories, themes, sub-themes, and example quotes.

Category	Themes	Sub-themes	Example quotes
Coaches' perceived levels and importance of physical activity	Athlete physical activity during training is important		“Yeah because if they get too many drink breaks they shut off, they're not motivated, they're not active, and they talk. Then the training session just drags out and doesn't become a good training session.” [SC 24].
			“The more you keep them active at training the easier it'll be coping in game situations when they're under pressure in the final quarter because they'll have that fitness. So, you know, it's really really important for them, far more than the club player who may only play a quarter or two.” [NC 23].
			“…at the beginning of the season they're a lot more active and we do a lot more running than they would later in the season later.” [SC 6].
	Athlete physical activity during training is not important		“I'd rather they be focused and lazy than running around not listening at all. I think that's more important… I've got to get across what we're trying to do – the skills and how we'll implement that in a game.” [NC 16].
	Training planning		“I wing it. I've been coaching for so many years I just make it up as I go.” [NC 14].
			“I write down what I want at the beginning of the year, but no, I don't write a formalised plan for each session it's more of a general idea.” [BC 11].
			“….the less committed the team is the less time I put into making a training session.” [BC 27].
	Athlete physical activity outside of orgnanised youth sport is important		“…anything they can do outside netball is only going to improve performance and make things easier during netball. So, that is important to me but I can't demand it and I don't initiate conversations about be active outside netball.” [NC 23].
			“Nowadays what we do as coaches is not enough because the kids aren't doing anything outside of the sports they play.” [BC 21].
			“For rep players it's important.” [BC 22].
			“If you want to play at an elite level, one 2-hour training session a week is not going to get you there.” [BC 19].
	Athlete physical activity outside of orgnanised youth sport is not important		“I believe that people should be active, especially kids, during and outside of sports. But, with the team that I'm coaching now, if I could get them all to training and get them to come to the game, that's two activity sessions a week and I'd be satisfied with that. If I was coaching a rep team, I'd expect them to do more than that.” [NC 8].

SC = soccer coach; NC = netball coach; BC = basketball coach.

**Table 6:** Coaches' perceptions on improving athlete physical activity: summary of categories, themes, sub-themes, and example quotes.

Category	Themes	Sub-themes	Example quotes
Coaches' perceptions on improving athlete physical activity	Perceives a need to increase athlete physical activity during training		“…there probably is a need to increase activity, but it might be hard to convince the girls.” [NC 17]
	Does not perceive a need to increase athlete physical activity during training		“No there's no need, I'm fairly happy with where we're at. I've been doing this for a while.” [BC 19].
	Methods to increase physical activity during training	Coach-specific methods	“Make sure that you're prepared and organised and that you set out a specific training schedule so that there isn't any down time.” [BC 21].
			“focus more on constant running or movement and less standing time, less watching, less waiting, and less listening to instructions from myself….” [BC 30].
		Drill modification	“…using modified drills. So, smaller groups and lots of equipment so they're really just keep chugging through.” [NC 13].
	Perceived responsibility to influence physical activity outside of organised youth sports		“No, I don't think I'm responsible for the girls outside of the sport… I don't have that much of an influence outside of soccer.” [SC 4].
			“With the rep players we encourage them to do things outside of netball but not with the club players.” [NC 23].
			“I don't feel a responsibility, but I'll use the word opportunity again, I think there's a huge opportunity as a coach.” [BC 29].
	Coach has the ability to impact health behaviours		“…I think I can because coaches I've had have had an impact on me and my sisters as well, I think I can….” [NC 7].
	Coach does not have the ability to impact health behaviours		“We [as coaches] only see the kids twice a week, once at training and once at the game, so I think parental influence is far outweighing anything I can do as a coach.” [NC 15].
			“…because I only see them for probably 2 hours a week I think other influences like parents, schools, and even friends would play a much larger role in influencing their physical activity.” [NC 16].

SC = soccer coach; NC = netball coach; BC = basketball coach.

**Table 7:** Coaches' perceived challenges: summary of categories, themes, sub-themes, and example quotes.

Category	Themes	Sub-themes	Example quotes
Coaches' perceived challenges	Coaches' perceived personal challenges	Time commitment to coaching	“There's a high level of commitment required in coaching you have the campaign, training, match day, phone calls and emails to organise everyone, etcetera, etcetera. It can be pretty time consuming.” [SC 4].
			“After having a whole shift at work all day and then having to organise the drills and getting them down-pat that's one barrier for me because this is my first year coaching.” [SC 9].
		Weak in some coaching aspect	“I'm good at the coaching and the motivating and leadership skills; but the technical skills is not my expertise, you know, I haven't really played a lot of soccer.” [SC 5].
			“ One of my weaknesses is getting kids focused when they need to be focused. When I was a younger coach, kids were having fun but they weren't actually getting better because there would be no focus at training.” [BC 27].
			“I'm coaching the kids based on my own experiences, you know, I haven't had any formal training so, that's a big barrier for me.” [SC 28].
		Work commitments	“I'm really really busy with work and I really try hard just to find the time to put the effort into being with the girls but often I have to get someone else to run training because I can't make it.” [SC 10].
	Coaches' perceived challenges relating to their athletes	Athletes' variability in skill/experience	“I suppose one of the big barriers I have with the 11's is that there is such a wide array of skill and experience. So, I have some girls that are really, really advanced and you have some that aren't, like I've got two girls playing their first year of netball. So, it's hard trying to catch them up as well as making the ones who want to advance not bored.” [NC 12].
		Athletes' lack of interest/focus	“…they do chatter a lot and that can be a problem sometimes, to keep them interested and keep them focused on what they're meant to doing.” [SC 10].
		Athletes' lack of motivation/commitment	“…lack of motivation is a barrier sometimes. Sometimes the girls probably don't take it as seriously as they should and some girls just see training as a social thing; which it definitely can be. But, it's important that they make an effort to train hard otherwise why bother coming?” [BC 30].
		Athlete management	“Sometimes the girls don't listen to what I tell them to do, like if I tell them to do warm up laps they'll complain and it becomes a negotiation, which wastes time.” [NC 17].
			“There's always one or two in most teams where you'll find a personality where you've got to work really hard to work out where they're coming from or what their problem is without having them blow up or getting upset or whatever. It's definitely an obstacle – one that you don't need.” [NC 23].
			“I've got one girl who hasn't spoken all year and one who is deaf so, she can't get instructions from me. With those girls in particular, it's been very difficult for me.” [SC 5].
	Coaches' perceived challenges relating to their athletes' parents	Managing parental expectations/perceptions	“…dealing with the parents is a big one… playing time; expectations on the teams' performance; their opinions on where I should be playing their daughter; parents who are yelling at refs, opposing parents, players… you name it.” [SC 3].
		Parental commitment	“The main barrier is getting the children to training. That's the main barrier. All the children like to play and as a general rule you'll get the children there on a Saturday to play, but the lack of commitment by the parents to get their kids to training is huge” [NC 8].
	Coaches' perceived challenges relating to promoting physical activity.		“There's just not enough time to do anything besides basketball. We only have two sessions a week for two hours.” [BC 21].

SC = soccer coach; NC = netball coach; BC = basketball coach.

### Perceived role as coaches

Coaches described roles in which they could be influential to their athletes, such as being a mentor or role model. The most common influential perceived role that coaches cited, though, was as a teacher:

*“Mainly I’m like a teacher and that’s what I want to be seen as because that’s what I’m doing - teaching the girls about netball… skills, strategy and so on.” [Netball coach 13].*

Within this theme, coaches described the need to foster sports-related development, promote the development of life skills, and to create a positive environment for their athletes. Sport-specific development was the focal point for many coaches, with a particular focus on teaching athletes skills, tactical/strategic awareness, and preparedness relevant to their sport. Another predominant topic discussed by coaches was their efforts to try to teach life skills through sport. The most frequently discussed life skills were accountability, confidence, respect, and social skills. Many considered generating a positive team environment to be an important aspect of their role as a coach. In particular, coaches identified the need to create an environment that was fun, friendly, and supportive.

Other coaches perceived their role to be that of a facilitator, which was described by coaches as someone who organises aspects of OYS (e.g., plan training sessions, set line ups, ensure equal playing time), or as a disciplinarian, which was described as someone who is strict and resolves conflicts amongst athletes. Perceived roles as a facilitator or disciplinarian, however, were not as common as the previously mentioned perceived roles.

### Coaches' perceptions of themselves as role models for PA

When asked, most coaches thought of themselves as a role model for PA, but many had not considered it before.

*“I suppose I haven't thought about it before now…. But, I think it's [being a role model] a given, you know, it's just an understanding you have, that if you're coaching and you're still playing they'll look up to you.” [Soccer coach 5].*

Other coaches cited their participation at training, their current involvement in the sport (as an athlete in a team), a physically active lifestyle, and their age and longevity in the sport as reasons for perceiving themselves as role models for PA for their athletes.

While most coaches considered themselves role models for PA, the view was not shared by all coaches. Poor fitness levels, old age, injury or health problems, and retirement from organised sports were the most common reasons for coaches not perceiving themselves as role models. Although some coaches did not perceive themselves as particularly good role models for the reasons listed above, some recognised the importance and the opportunity they had to be role models.

*“I see the importance of people like me being a role model for our players… the truth is you don't have to be a physically fit person to inspire others to be fit. But, role modelling is always important and there is an opportunity as coaches to be a fantastic role model.” [Basketball coach 29].*

### Perceived levels and importance of PA

#### Coaches' perceived importance related to athletes' PA during training

Coaches' perceptions relating to the importance of athlete PA during training were not universal. The majority of coaches, however, perceived PA to be important during training, with some stating that being physically active is more important to them than winning.

*“…keeping the girls active at training is very important, it's one things I really try to do. I love seeing the girls improve their fitness, their skills… and hey, if we get some wins along the way, that's great too (laughs).” [Basketball coach 11].*

Some coaches mentioned that a physically active training session was needed to keep girls motivated and engaged. Other coaches stated that the athletes would benefit by being physically active during training because their fitness levels will allow them to outperform their opposition late in games.

Also, a few coaches discussed how they front-loaded their training sessions to include higher intensity PA at the beginning of the season and purposefully dropped the PA intensity at training as the season went on. The reason that coaches did this was because they felt girls' fitness levels were not maintained over the off-season, so the focus of training sessions at the beginning of the season was to regain girls' fitness. Once coaches felt the girls' fitness was regained, the focus of their training sessions shifted to skill development, where coaches perceived PA intensity to drop.

*“Early in the year, fitness training was huge because the girls were pretty low in fitness, you know, they had the summer holidays and they hadn't done much. But, as we move on during the season, ball skills and controlling the ball become paramount… then it's lots of drills and getting their positions right. So the intensity at training drops a bit because we do more drills and focus less on the fitness aspect.” [Soccer coach 9].*

Coaches who felt that their athletes' PA level during training was not important tended to believe that it was more important to focus on teaching sport-related skills and skill development. These coaches were willing to sacrifice PA intensity to achieve this.

#### Perceived levels of PA

Most coaches felt that they were conscious of their athletes' PA levels and that they were able to gauge how active the girls were at training. Furthermore, the majority of coaches considered high intensity PA to be inherent in OYS.

*“I'm always on them about different things, trying to keep the intensity up… and as a coach you can gauge how the team is training … so, if the group is down then I can quickly gauge that the intensity is down and I'll try to pick it up.” [Basketball coach 20].*

*“…I try to keep the girls moving and high intensity activity is natural in soccer.” [Soccer coach 1].*

#### Training session preparation

Coaches' training preparation responses were highly variable, ranging from developing a meticulously written training plan to no planning at all. In this sample of coaches, very few coaches actually wrote down their plan for training, with many claiming that they just mentally prepare for their training sessions.

*“I usually just plan in my head on my way to training, so it's mentally written down… so, there is the warm up that I want to do, there are certain drills I want to do and there is a cool down….” [Netball coach 12].*

Some coaches discussed having general or thematic (e.g., shooting drills, passing drills) training session plans in mind rather than including specific drills, claiming that they are experienced enough to come up with specific drills on-the-spot. Some even claimed that they would just “wing it” during their training sessions, relying on their coaching experience to develop a session as-they-go. Some coaches with multiple teams admitted that they spent less time preparing training sessions for their less competitive teams. The majority of coaches said that their focus at training was based on observed weaknesses from the previous game.

#### Coaches' perceived importance related to athletes' PA outside of OYS

Athletes' PA outside of OYS was perceived as being important by most coaches. This was due to the perceived positive effect it would have on performance in OYS. Also, being physically active outside of OYS was perceived as being more important for representative athletes compared to club athletes by coaches; especially if there was a desire to play at an elite level. It appeared that coaches were content if club athletes attended their weekly training session and game, but for representative athletes the expectation to be physically active went beyond weekly training and games; these athletes were expected to be physically active in some way outside of OYS.

Some coaches reflected on changes in norms from their childhood where playing outside was regarded as a norm, compared to now where coaches perceive children to be doing very little outside of OYS.

*“I remember when I was a kid, you get home from school, you go down to your mate's place and play basketball, footy, soccer, whatever, or you're on your push bike… now you don't see any push bikes or anything like that. It's a completely different lifestyle than when I was a kid. [Basketball coach 21].*

*“It's not like it used to be back when I was a kid, we used to play outside until it got dark every night after school. Things have changed and I think that the kids have got to do something outside of your training session to get better, I think a lot of kids today come to training and that's it for the week.” [Basketball coach 29].*

### Coaches' perceptions on improving athlete PA

#### Perceived need to increase athlete PA during training

Few coaches perceived the need to increase PA because they were content with the level of PA during their training sessions. Some coaches, however, reported having to reduce the intensity of their training sessions because of the girls' disinclination to train at a high intensity.

*“…the girls were just not keen to put the effort into the training sessions that I was running…. I've had to re-adjust my focus and my expectations for the girls and I'm happy where we sit now with the level of activity” [Soccer coach 2].*

A major concern raised by coaches was a fear of athlete dropout if the PA intensity during training in OYS was too high.

*“You can't push some of these girls too much, because they'll quit. You can try to be motivational to get them to be more active, but you can't force them, you know.” [Basketball coach 22].*

*“…there's a lack of fitness in probably two-thirds of the side and there's a reluctance to put the effort in…. So, if I were to step up the intensity, there would be more of a dropout rate. A lot of the girls fake injury to sit out as it is.” [Soccer coach 4].*

*“…they would revolt [if the coach tried to increase PA]. They would just go ‘no, I'm not doing it’ or they wouldn't come to training. So, you've really got to gauge how far you can push them. [Netball coach 15].*

One coach, however, emphasised the need to take advantage of the time spent in OYS because she has noticed that the girls who she coaches are less active and has noticed changes in body shape and their physical ability.

*“…compared to 10 years ago, the girls I coach are generally less active, and I've noticed that they don't have the same gross motor skills as they would've had 10 years ago. I definitely see a change in body shape and physical ability. So, I think we need to take advantage of the time kids are at basketball because for some, this is all the activity they get in a week.” [Basketball coach 21].*

#### Methods to increase PA during training

Although most coaches did not feel the need to increase PA during their training sessions, they were, however, able to identify ways to increase training session PA if they needed to. Coaches suggested improving their organisation, increasing preparation for training, developing more specific training plans, and reducing waiting (i.e., in lines during drills or during drill tranisition) and instruction time. They also suggested modifying drills to include smaller groups and having more equipment available.

#### Perceived responsibility to influence PA outside of OYS

Although most coaches felt that their athletes should be physically active outside of OYS, very few felt it was their responsibility to influence PA outside of OYS. Coaches felt that they had very little influence over their athletes' PA behaviours outside of OYS, most commonly citing parents as more influential in this respect. Peers were also considered by coaches to have a greater influence on PA levels outside of OYS than they did.

The comparison between representative athletes and club athletes emerged once again while discussing coaches' perceived responsibility to influence PA outside of OYS. Some coaches thought it was more likely that they could encourage representative athletes to train in their free time outside of OYS as opposed to club athletes; however, this was seldomly discussed.

Although not feeling a responsibility to influence PA outside of OYS, some acknowledged that coaches in OYS have a substantial opportunity to do so. See Table 6 for supporting quotes.

#### Coaches' perceived ability to impact health behaviours

When coaches were asked if they felt they had the ability to impact girls' health behaviours, coaches took a very pragmatic approach. Some coaches stated they have had coaches that have had a lasting impact on them, so it was plausible that they could have a lasting impact on their athletes. There were no identifible charateristics that were apparent among coaches with differing opinions of their perceived ability to impact girls' health behaviours (i.e., sport coached, coach's gender, coaching experience).

Interestingly, PA was rarely discussed as a health behaviour when identifying whether coaches thought they could impact their athletes' health behaviours or not. Often the conversation shifted from the designed focus on PA to coaches discussing their attempts to inform their athletes about healthy eating.

*“I try to encourage healthier eating, like I had one girl that used to eat a meat pie before a game, so I tried to get her in the habit of eating the correct foods before games. That's one area where I think I can leave an impression…. what they eat and how they prepare is important and I think I can help with that.” [Netball coach 18].*

Most coaches, though, perceived their ability to impact girls' health behaviours was limited. Insufficient exposure and influence were the main reasons that coaches could not impact girls' health behaviours. Again, parents, teachers, and peers were considered to have a greater influence on girls' health behaviours.

### Coaches' challenges in OYS

#### Coaches' perceived personal challenges relating to OYS

Few coaches felt they had any personal challenges while coaching in OYS. The perceived time needed to commit to OYS was, however, the main issue identified by coaches who did report having personal challenges. The time needed for administrative tasks as well as preparing for training were the two biggest time consumers, with the latter particularly affecting less experienced coaches. Some coaches discussed an over-commitment to their sport; this included coaching and refereeing multiple teams and games, respectively.

*“Maybe an over-commitment to basketball… I can only be in one place at one time and sometimes it clashes with training. It takes a toll on you, some nights I'm coaching non-stop.” [Basketball coach 20].*

*“…Friday nights I'm here coaching three teams and reffing two, so it's just bang-bang-bang five games in a row.” [Basketball coach 25].*

Some coaches felt that they were weak in some aspects of coaching, which they perceived as a limitation in their coaching ability. Perceived coaching weaknesses included poor sport-specific technical skills, difficulty keeping athletes focused on the task at hand, and lack of formal training. Work commitments also emerged as an issue faced by coaches occasionally, but were not commonly discussed.

#### Coaches' perceived challenges relating to their athletes

A predominant challenge coaches discussed was the wide variation in athletes' skill levels and experience within a team. Some coaches described the dilemma of trying to find the right balance at training, where the skilled/experienced athletes feel engaged without leaving the less skilled/experienced athletes to fall further behind.

Girls' focus and interest levels posed problems for coaches as well, with the main reported obstacle being that girls talk too much during training. Some coaches described training as a “social gathering” and felt that girls' motivation and commitment was lacking. As a negotiation with the girls, some coaches have implemented “talk time” where they are allowed to talk at certain points of the training session, in an effort to minimise conversations that are not sports-related.

*“I've had to implement, what I call, ‘talk time’ to keep the conversations to a minimum during training… see a lot of them went to primary school together and they're at different high schools. So, it's like a reunion every Wednesday night.” [Soccer coach 9].*

Athlete management was another theme that emerged as an athlete-related challenge, which related to non-compliance with coach instructions, difficult athletes, and athletes with disabilities. See Table 7. for supporting quotes.

#### Coaches' perceived challenges relating to their athletes' parents

All coaches, at one point or another, experienced some sort of issue relating to their athletes' parents during their years coaching OYS. Athletes' playing time was one of the most common complaints from parents. Parental commitment to OYS was cited as a major issue for coaches as well, with the main perceived issue being parents' unreliability when it came to getting their daughters to training.

Also, one coach was frustrated with some parents' lack of interest in the sport that their daughter was playing and felt that the lack of parental support could impact on further participation in OYS.

*“It annoys me when the parents aren't quite on the same wavelength as you because I love this stuff [netball], okay, and I think most of the girls do too. So, it bothers me when parents don't take any interest in it and I'd bet there are probably kids who stop playing netball because they don't have any support from their mum or dad.” [Netball coach 13].*

Another coach noticed that, as the girls on his team got older, fewer parents were attending their daughters' training and game sessions.

*“When I started coaching them at 12… all the parents were there and now, no parents are there.” [Soccer coach 1].*

#### Coaches' perceived challenges relating to promoting PA

Frequency and duration of training sessions were the most commonly cited challenges with regard to promoting PA. Coaches felt they had too little time at training to discuss anything outside of the sport they were coaching.

## Discussion

To our knowledge, this is the first study to explore whether coaches perceive themselves as influential on PA for girls participating in OYS. More specifically, we explored coaches' perceived role as coaches, their perception of themselves as role models for PA, their views on their athletes' current PA levels, their opinions on improving their athletes' PA levels, and their perceived challenges during OYS. Our analysis of 30 in-depth semi-structured interviews suggests that most coaches feel that they have the potential to influence PA for girls in OYS. It is possible, though, that coaches may underestimate or not fully realise the impact they can have on the girls they coach in OYS.

When asked about their perceived role as a coach, a range of influential roles were discussed. The perception of being a teacher, role model, or mentor resonated with many of the coaches in this study. The fact that several influential roles resonated with coaches is a positive finding from a PA promotion standpoint, as Smith and Smoll [4] have suggested that coaches can have a strong impact on children and adolescents due to consistent direct involvement with them. Not surprisingly, coaches primarily reported that it was their responsibility to provide sport-specific development (e.g., technical skills, tactical awareness, preparedness). Coaches also reported, however, that it was part of their role to create a positive environment (e.g., fun, friendly, supportive) and to foster the development of life skills, which was also found in recent study by Vella et al. [32]. Those authors also noted that the responsibility coaches felt to develop athletes' life skills was an important extension to existing literature and our study lends support to that finding.

While some coaches had never considered it before the interview, the majority perceived themselves to be role models for PA, particularly if they were still currently involved in organised sports in some capacity (i.e., active participants during training or currently playing in a team). Although no direct comparisons are available, Drummond et al. examined student and health educators' perceptions in relation to role modelling exercise [29]. The authors found that 90% (18 out of 20) of health educators perceived themselves as role models for exercise for their students, citing their participation level as the main reason for this perception [33]. In contrast to our findings, however, nonparticipation in sports was not cited as a reason for health educators not perceiving themselves as role models for exercise in the study by Drummond et al. [33].

Most coaches stated that being physically active during OYS was important. Coaches reported that they were conscious of their athletes' PA levels and had the ability to gauge their athletes' PA levels. The presumption by many, however, was that high-intensity PA was inherent to OYS. So, it is not surprising that most coaches felt it was unnecessary for them to try to increase girls' PA levels and reduce their inactivity during training. Smith and Smoll's [4] research, however, indicates that coaches have limited awareness of their actions during OYS and state that increasing awareness is essential for change to occur. Therefore, low-cost methods, such as pedometers or direct observation systems (e.g., the System for Observing Fitness Instruction Time [34]), could be used to provide coaches with objectively measured feedback on girls' PA levels, and self-monitoring could be introduced to coaches in an effort to assist in optimising time spent in training during OYS.

An interesting theme that emerged was the concern held by coaches that girls might drop out of OYS if, for a prolonged period training, PA intensity was too high. Coaches' recognition that they could be responsible for prompting athletes' withdrawal is a positive finding. Youth athletes in other studies have ranked their coach as the most influential person in making the decision to withdraw from OYS [35], where one study found that coaches influenced nearly one-third of athletes to withdraw from OYS [36]. Of the extensive literature that exists relating to athlete dropout from OYS [37]–[39], as far as we are aware, high-intensity PA is not commonly reported as a reason for withdrawal from OYS among athletes. One study sampled nearly 400 athletes and reported over 30 reasons for athlete withdrawal from OYS and none of the athlete-reported reasons related specifically to PA intensity. This is not to say that high-intensity PA cannot influence girls' decision to withdraw from OYS. Though, as far as we are aware, coaches' perception that girls may withdraw from OYS due to high intensity PA does not appear to be in line with athlete-reported reasons for dropping out of OYS. Further exploration on this topic is warranted and should be taken into consideration in any PA promotion interventions in OYS involving girls.

Generally, coaches in this study reported spending little time preparing for training sessions. The majority of coaches said that they relied on their experience to create impromptu training sessions. Mandic and colleagues have suggested that coaches should ensure that training session drills are structured to maximise PA intensity [40]. Further supporting a structured training session, a recent study conducted in a physical education setting found a negative correlation between time spent in management (i.e., drill transition, instruction) and student MVPA [23]. Without prior preparation, there is a greater likelihood that time at training is not being used as efficiently as it can be, and PA intensity could potentially drop.

Coaches reported that they were capable of altering their training sessions to increase girls' PA, if they felt they needed to. Coaches were able to identify numerous strategies that could be employed in their training sessions to increase opportunities to be active, reduce inactivity, and improve their efficiency and management of training. Many of the strategies that coaches identified have also been recommended within a physical education setting; and included: using smaller groups, providing more equipment, reducing waiting, and reducing instruction time to increase girls' opportunities to be physically active [41], [42]. However, coaches' awareness of these strategies may not necessarily mean they will employ them because knowledge can be a poor predictor of behaviour [43]; especially if coaches' perception of girls' PA during training is already considered adequate. Approaches are needed, then, to ensure that coaches are not only aware of strategies to increase opportunities to be active (and reduce inactivity), but also have the belief that as a result of implementing these strategies it can lead to positive outcomes (e.g., health benefits) [43].

Most coaches stated that being physically active during OYS was important, however, rarely discussed the health benefits associated with being physically active. Coaches in this study felt confident discussing the sport they coached, but may lack confidence discussing the more general health benefits associated with PA. Coaches' perceived ability to impact girls' health behaviours was also discussed, and few coaches felt that they could have an impact on the health behaviours of the girls they coached. This belief may represent a missed opportunity for coaches to make a meaningful impact on girls' health behaviours as girls can learn behaviours from their coaches, particularly if the girls admire their coach [44]. Coaches did not feel that they were able to impact their girls' health behaviours, and two of the main reasons for this were a perceived lack of influence and limited exposure to their athletes. However, Smith and Smoll [4] suggest the contrary, coaches can greatly impact their athletes. Interestingly, PA was rarely mentioned as a health behaviour that coaches felt they could impact, rather healthy eating was commonly discussed instead. This may be due to coaches' perception that PA is inherent to OYS.

Outside of OYS, coaches discussed changes in norms from their childhood where unstructured leisure-time PA was regarded as a norm. They also perceived there to be a decline in PA amongst children and adolescents, however, very few coaches felt responsible for influencing girls to be physically active outside of OYS. Even though most coaches perceived their role to be one that could be influential to their athletes in OYS, it appears many of them do not perceive their influence to extend outside of OYS. Coaches suggested that parents and peers had a greater influence on PA outside of OYS than coaches did. There is ample evidence to support coaches' claims that parents and peers are influential in supporting children to be physically active [45]–[47]; however, one study found that physical education teachers were as influential as parents in supporting adolescents' PA outside of school [48]. While this is not a direct comparison, it is possible that OYS coaches can also greatly influence girls' PA outside of OYS and coaches are underestimating the impact they can have.

The most commonly perceived personal challenge experienced by coaches was the amount of time they felt they needed to commit to OYS. Administrative tasks and preparing for training were considered the two biggest perceived consumers of coaches' time. Many coaches, however, stated that they relied on their experience to plan training sessions somewhat spontaneously. Coaches also identified a number of challenges relating to coaching their athletes. The predominant issue was the amount of variation in skill level and experience within their teams. Some coaches found it difficult to keep the skilled/experienced girls engaged during training without having the less skilled/experienced girls falling further behind, likely increasing the amount of instruction needed. These findings could potentially result in training sessions that do not maximise athletes' opportunities to be physically active. These are important findings as previous literature has shown that for the majority of time during OYS athletes are inactive or in light PA [12], [13], [21], [22]. Furthermore, Dudley et al. [23] found negative correlations between instruction/management and MVPA. This valuable insight could inform future studies aiming to increase PA in OYS.

Coaches also reported girls' focus/interest levels, motivation/commitment, and athlete management as challenges. Although coaches identified these as challenges, they seemed confident in their ability to deal with them, often detailing how they overcome them.

When coaches discussed their perceived challenges in relation to parents, an interesting finding from a PA promotion perspective was that some coaches believed that they were able to identify girls on their teams who had low parental support. Coaches reported being frustrated with some parents' lack of commitment and support for their daughters. A coach commented on how annoyed she was with parents who did not take any interest in the sport their daughter played, and suggested that girls with a lack of parental support are likely to stop playing OYS. This is an encouraging finding as there is strong evidence to suggest that parental support is linked with children's PA behaviours [49]–[52] and children's participation in OYS [53], [54]. Furthermore, Lubans, Sylva, and Morgan [55] found that in older adolescents, parental support was significantly correlated with MVPA; however, one coach commented on his observation that parents' presence during OYS has decreased as the girls he coached got older. Given that girls' PA levels tend to decrease sharply in adolescence [17], [19], maintaining parental support may be an important factor to consider in efforts to increase and maintain PA levels in girls as they transition into adolescence and adulthood. As coaches in this study were able to identify athletes lacking this much-needed parental support, coaches may be able to play an important role maintaining parental support and should be examined further.

Some potential limitations should be considered when interpreting these findings. Firstly, it is possible that coaches offered socially desirable viewpoints during their interview. Secondly, a convenience sample was used, possibly introducing an element of selection bias. That said, a wide array of responses from a diverse sample of coaches was collected. Lastly, female-coaching perspectives may be underrepresented as our sample contained more men than women; however, male coaches are more prevalent than female coaches in OYS [56]. Despite these limitations, the present study provides unique insight into coaches' perceptions of themselves as being influential on PA for girls in OYS. Also, rigorous research methodology was employed to ensure the trustworthiness of the data. We used several strategies [57] to strengthen the credibility of our data, for example, investigator triangulation during the interpretation phase, individual classification during data analysis, reflexivity, and member checking. Along with aiding in the credibility of the data, the abovementioned strategies also protected against individual perceptual biases [58]. According to Lincoln and Guba [59], demonstrating credibility may be considered sufficient to support the notion of dependability. Further, we have established acceptable confirmability by using published guidelines to analyse our data [29], [31] and, as mentioned above, employed strategies to reduce individual perceptual biases. Lastly, concerning transferability, Lincoln and Guba [59] suggested that transferability is primarily the responsibility of the researcher interested in transferring the findings to another context or population than that of the original study. Lincoln and Guba [59] also state that so long as the original study presents sufficient descriptive data to allow comparisons the issue of transferability has been adequately addressed. The current study provided a thorough description of the research context and adequate descriptive data allowing other researchers to make judgement on how practical a transfer of the results are to a different context or population.

Considering the high proportion of children that participate in OYS, and the myriad of health and developmental benefits associated with the setting, OYS has the potential to be a powerful health-promoting environment for children and adolescents. Recently a number of studies have examined OYS clubs as a setting to promote health [9], [10], [60]. These studies illustrate a wide range of health-promoting capabilities OYS can provide and the importance of OYS clubs. However, only one study recognised that OYS clubs can play a role in promoting PA [60]. Our study provides a unique perspective on OYS coaches' perceptions of themselves as being influential on PA for girls in OYS. Further, coaches in this study (whilst not the primary focus) indicated that they were confident discussing healthy eating with the girls on their team. They may, however, underestimate or not fully realise the impact they can have. To further enhance the health-promoting capabilities of OYS, there should also be an emphasis placed on educating coaches to capitalise on the opportunity they have to promote PA to the girls they coach. This information on OYS can be used as a platform on which to inform policies, programs, and interventions to develop strategies to increase girls' PA levels through OYS.
